# Stroke Disease Detection and Prediction Using Robust Learning Approaches

**DOI:** 10.1155/2021/7633381

**Published:** 2021-11-26

**Authors:** Tahia Tazin, Md Nur Alam, Nahian Nakiba Dola, Mohammad Sajibul Bari, Sami Bourouis, Mohammad Monirujjaman Khan

**Affiliations:** ^1^Department of Electrical and Computer Engineering, North South University, Bashundhara, Dhaka 1229, Bangladesh; ^2^Department of Information Technology, College of Computers and Information Technology, Taif University, P.O. Box 11099, Taif 21944, Saudi Arabia

## Abstract

Stroke is a medical disorder in which the blood arteries in the brain are ruptured, causing damage to the brain. When the supply of blood and other nutrients to the brain is interrupted, symptoms might develop. According to the World Health Organization (WHO), stroke is the greatest cause of death and disability globally. Early recognition of the various warning signs of a stroke can help reduce the severity of the stroke. Different machine learning (ML) models have been developed to predict the likelihood of a stroke occurring in the brain. This research uses a range of physiological parameters and machine learning algorithms, such as Logistic Regression (LR), Decision Tree (DT) Classification, Random Forest (RF) Classification, and Voting Classifier, to train four different models for reliable prediction. Random Forest was the best performing algorithm for this task with an accuracy of approximately 96 percent. The dataset used in the development of the method was the open-access Stroke Prediction dataset. The accuracy percentage of the models used in this investigation is significantly higher than that of previous studies, indicating that the models used in this investigation are more reliable. Numerous model comparisons have established their robustness, and the scheme can be deduced from the study analysis.

## 1. Introduction

Stroke occurs when the blood flow to various areas of the brain is disrupted or diminished, resulting in the cells in those areas of the brain not receiving the nutrients and oxygen they require and dying. A stroke is a medical emergency that requires urgent medical attention. Early detection and appropriate management are required to prevent further damage to the affected area of the brain and other complications in other parts of the body. The World Health Organization (WHO) estimates that fifteen million people worldwide suffer from strokes each year, with one person dying every four to five minutes in the affected population. Stroke is the sixth leading cause of mortality in the United States according to the Centers for Disease Control and Prevention (CDC) [1]. Stroke is a noncommunicable disease that kills approximately 11% of the population. In the United States, approximately 795,000 people suffer from the disabling effects of strokes on a regular basis [2]. It is India's fourth leading cause of death. Strokes are classified as ischemic or hemorrhagic. In a chemical stroke, clots obstruct the drainage; in a hemorrhagic stroke, a weak blood vessel bursts and bleeds into the brain. Stroke may be avoided by leading a healthy and balanced lifestyle that includes abstaining from unhealthy behaviors, such as smoking and drinking, keeping a healthy body mass index (BMI) and an average glucose level, and maintaining an excellent heart and kidney function. Stroke prediction is essential and must be treated promptly to avoid irreversible damage or death. With the development of technology in the medical sector, it is now possible to anticipate the onset of a stroke by utilizing ML techniques. The algorithms included in ML are beneficial as they allow for accurate prediction and proper analysis. The majority of previous stroke-related research has focused on, among other things, the prediction of heart attacks. Brain stroke has been the subject of very few studies. The main motivation of this paper is to demonstrate how ML may be used to forecast the onset of a brain stroke. The most important aspect of the methods employed and the findings achieved is that among the four distinct classification algorithms tested, Random Forest fared the best, achieving a higher accuracy metric in comparison to the others. One downside of the model is that it is trained on textual data rather than real time brain images. The implementation of four ML classification methods is shown in this paper.

Numerous academics have previously utilized machine learning to forecast strokes. Govindarajan et al. [3] used text mining and a machine learning classifier to classify stroke disorders in 507 individuals. They tested a variety of machine learning methods for training purposes, including Artificial Neural Network (ANN), and they found that the SGD algorithm provided the greatest value, 95 percent. Amini et al. [4, 5] performed research to predict a stroke occurrence. They classified 50 risk variables for stroke, diabetes, cardiovascular disease, smoking, hyperlipidemia, and alcohol consumption in 807 healthy and unhealthy individuals. They used two of the most accurate methods: the c4.5 decision tree algorithm (95 percent accuracy) and the K-nearest neighbor algorithm (94 percent accuracy). Cheng et al. [6] presented a study on estimating the prognosis of an ischemic stroke. In their study, they used 82 ischemic stroke patient data sets, two ANN models, and the accuracy values of 79 and 95 percent. Cheon et al. [7–9] conducted research to determine the predictability of a stroke patient death. They identified the stroke incidence using 15,099 individuals in their research. They detected strokes using a deep neural network method. The authors utilized PCA to extract information from the medical records and predict strokes. They have 83 percent area under the curve (AUC). Singh et al. [10] conducted research using artificial intelligence to predict strokes. They employed a new technique for predicting stroke in their research using the cardiovascular health study (CHS) dataset. Additionally, they used the decision tree method to do a feature extraction followed by a principal component analysis. In this case, the model was built using a neural network classification method, and it achieved 97 percent accuracy.

Chin et al. [11] conducted research to determine the accuracy of an automated early ischemic stroke detection. The major objective of their research was to create a method for automating primary ischemic stroke using Convolutional Neural Network (CNN). They amassed 256 pictures for the purpose of training and testing the CNN model. They utilized the data lengthening technique to increase the gathered picture in their system's image preparation. Their CNN technique achieved a 90 percent accuracy rate. Sung et al. [12] conducted research to establish a stroke severity index. They gathered data on 3577 patients who had an acute ischemic stroke. They utilized a variety of data mining methods, including linear regression, to create their predictive models. Their ability to predict outperformed the k-nearest neighbor method (95% confidence interval). Monteiro et al. [13] used machine learning to predict the functional prognosis of an ischemic stroke. They tested this method on a patient who died three months after admission. They obtained an AUC value of greater than 90. Kansadub et al. [14] conducted research to determine the risk of stroke. The authors of the research analyzed the data to predict strokes using Naive Bayes, decision trees, and neural networks. They assessed their pointer's accuracy and AUC in their research. They categorized all of these algorithms as decision trees, with naive Bayes providing the most accurate results. Adam et al. [15] conducted research to determine the classification of an ischemic stroke. They categorized ischemic strokes using two models: the k-nearest neighbor method and the decision tree technique. In their study, the decision tree method was found to be more useful by medical experts when used to categorize strokes.

The majority of studies had an accuracy rate of around 90%, which was considered to be quite good. However, the novelty of our research is that we used several well-known machine learning methods to get the best result. Random forest (RF), decision tree (DT), voting classifier (VC), and logistic regression (LR) were the most successful algorithms, with 96, 94, 91, and 87 percent F1-scores, respectively. The accuracy percent of the models used in this research is much greater than the accuracy percent of the models used in previous investigations, suggesting that the models used in this investigation are more trustworthy. They have been shown to be resilient in many model comparisons, and the scheme may be generated from the results of the study's analysis.

As mentioned earlier, the major contribution of this research is that we have used different machine learning models on a publicly available dataset. In the previous work, most of the researchers used a significant model to predict the stroke disease. However, we used four different models, and also, we compared the results with the previous work. All the results and comparisons are briefly discussed in the following section. The rest of this article is set out as follows: the experimental methodology and procedures are described in Section 2; the result analysis is provided in Section 3; and conclusions have been discussed in Section 4.

## 2. Procedure and Experimental Methodology

This section includes a description of the dataset, a block diagram, a flow diagram, and evaluation matrices, as well as the process and methodology used in the study.

### 2.1. Proposed System

The data has become available for model construction once it has been processed. A preprocessed dataset and machine learning techniques are needed for the model construction. LR, DT classification, RF classification, and voting classifier are some of the methods used. After creating four alternative models, the accuracy measures, namely accuracy score, precision score, recall score, and F1 score are used to compare them. The designed system's block diagram is shown in Figure 1.

All the components of the block diagram have been discussed in the following subsections.

### 2.2. Dataset

The stroke prediction dataset [16] was used to perform the study. There were 5110 rows and 12 columns in this dataset. The value of the output column stroke is either 1 or 0. The number 0 indicates that no stroke risk was identified, while the value 1 indicates that a stroke risk was detected. The probability of 0 in the output column (stroke) exceeds the possibility of 1 in the same column in this dataset. 249 rows alone in the stroke column have the value 1, whereas 4861 rows have the value 0. To improve accuracy, data preprocessing is used to balance the data.  Figure 2 shows the total number of stroke and nonstroke records in the output column before preprocessing.

From Figure 2, it is clear that this dataset is an imbalanced dataset. The SMOTE technique has been used to balance this dataset.

### 2.3. Preprocessing

Before building a model, data preprocessing is required to remove unwanted noise and outliers from the dataset that could lead the model to depart from its intended training. This stage addresses everything that prevents the model from functioning more efficiently. Following the collection of the relevant dataset, the data must be cleaned and prepared for model development. As stated before, the dataset used has twelve characteristics. To begin with, the column id is omitted since its presence has no bearing on model construction. The dataset is then inspected for null values and filled if any are detected. The null values in the column BMI are filled using the data column's mean in this case.

Label encoding converts the dataset's string literals to integer values that the computer can comprehend. As the computer is frequently trained on numbers, the strings must be converted to integers. The gathered dataset has five columns of the data type string. All strings are encoded during label encoding, and the whole dataset is transformed into a collection of numbers. The dataset used for stroke prediction is very imbalanced. The dataset has a total of 5110 rows, with 249 rows indicating the possibility of a stroke and 4861 rows confirming the lack of a stroke. While using such data to train a machine-level model may result in accuracy, other accuracy measures such as precision and recall are inadequate. If such an unbalanced data is not dealt with properly, the findings will be inaccurate, and the forecast will be ineffective. As a result, to obtain an efficient model, this unbalanced data must be dealt with first. The SMOTE technique was employed for this purpose.  Figure 3 depicts the dataset's balance output column.

The next stage is to construct the model after finishing data preparation and managing the imbalanced dataset. To improve the accuracy and efficiency of this job, the data is divided into training and testing data with a ratio of 80 percent training data and 20 percent testing data. After splitting, the model is trained using a variety of classification methods. Random forest, decision tree classification method, voting classifier, and logistic regression are the classification algorithms utilized in this study.

### 2.4. Proposed Algorithms

The most common disease identified in the medical field is stroke, which is on the rise year after year. Using the publicly accessible stroke prediction dataset, the study measured four commonly used machine learning methods for predicting brain stroke recurrence, which are as follows:

- Random forest
- Decision tree
- Voting classifier
- Logistic regression

#### 2.4.1. Random Forest

The classification algorithm chosen was RF classification [17]. RFs are composed of numerous independent decision trees that were trained individually on a random sample of data. These trees are created during training, and the decision trees' outputs are collected. A process termed voting is used to determine the final forecast made by this algorithm. Each DT in this method must vote for one of the two output classes (in this case, stroke or no stroke). The final prediction is determined by the RF method, which chooses the class with the most votes. A block diagram of random forest classification is shown in Figure 4.

The flexibility of the random forest is one of its most alluring features. It may be utilized for relapse detection and grouping tasks, and the overall weighting given to information characteristics is readily apparent. Additionally, it is a beneficial approach since the default hyperparameters it employs often give unambiguous expectations. Understanding the hyperparameters is critical since there are relatively few of them, to begin with. Overfitting is a well-known problem in machine learning, although it occurs seldom with the arbitrary random forest classifier. If there are sufficient trees in the forest, the classifier will not overfit the model.

#### 2.4.2. Decision Tree

Both regression and classification concerns are addressed using classification with DT [18]. Furthermore, as the input variables already have a related output variable, this methodology is a supervised learning model. It resembles a tree. The data is constantly segmented according to a specific parameter in this method. The decision node and the leaf node are the two parts of a decision tree. At the former node, the data is divided, and the latter is the node that produces the result. The DT classifier's basic structure is depicted in Figure 5.

The DT is easy to comprehend since it replicates the phases that a person goes through while making a real world decision. It may be very beneficial in resolving issues with decision-making. Consider all potential solutions to an issue. Cleaning data is not required as much as it is with other methods.

#### 2.4.3. Voting Classifier

A voting classifier is a type of classification model that trains on an ensemble of multiple models and predicts an output (class) based on the class that has the greatest chance of being selected as the output [19]. It is used to predict the outcome of a vote. The flowchart for the voting classifier model is shown in Figure 6.

Voting summarizes the methodology we will use to compare various training models. There are two methods of voting, which are as follows:

- Soft voting: In this phase, the predicted probability gradients for each model are added and averaged. The category with the highest value is deemed the winner, and its contents are the output. While this seems to be a fair and rational strategy, it is only recommended if the individual categories are calibrated correctly. This is similar to computing the weighted average of a set of numbers, except that each of the various models contributes proportionally to the final output vector.
- Hard voting: This phase combines the categorization outputs of all the various models and specifies the final output value as the mode value of the resultant output. Because of the fact that the particular probability values associated with each model are disregarded, this approach is analogous to computing the arithmetic mean of a collection of numbers. The output alone of each model is considered.

#### 2.4.4. Logistic Regression

The flowchart for the logistic regression model is shown in Figure 7. In the supervised learning approach, LR is one of the most commonly used ML algorithms [20]. It is a forecasting method that uses a collection of independent factors to predict a categorical dependent variable.

Utilizing logistic regression, the output of a categorical dependent variable is predicted. As a result, the output must be discrete or categorical in nature. It may be yes or no, 0 or 1, true or false, etc., but probability values between 0 and 1 are given. Logistic regression and linear regression are used in very similar ways. The classification problems are addressed with LR, and the regression problems are addressed using linear regression. Instead of a regression line, we use an S-shaped logistic function that predicts the two maximum values (0 or 1).

### 2.5. Evaluation Matrix

Figure 8 depicts the confusion matrix or evaluation matrix. The confusion matrix is a tool for evaluating the performance of machine learning classification algorithms. The confusion matrix has been used to test the efficiency of all models created. The confusion matrix illustrates how often our models forecast correctly and how often they estimate incorrectly. False positives and false negatives have been allocated to badly predicted values, whereas true positives and true negatives were assigned to properly anticipated values. The model's accuracy, precision-recall trade-off, and AUC were utilized to assess its performance after grouping all predicted values in the matrix.

## 3. Result Analysis

The models' capacities, model forecasts, investigation, and eventual outcomes are examined in this part.

### 3.1. Data Visualization

A histogram depicts a recurrence dispersion with infinite classes. It is a region outline made of square shapes with bases at class boundary spans and regions proportionate to the comparing classes' frequencies. As the base fills in the spaces between the class borders, the square shapes are all linked. The squares form the statures are proportional to the comparative class frequencies and recurrence densities for distinct classes.  Figure 9 illustrates some important features of the histograms. A histogram depicts the dataset's proportions.

Figure 9 depicts the dataset's gender, age, hypertension, heart disease, ever married, average glucose level, and body mass index distributions. For the gender attribute, 0 means male and 1 means female. There are more female samples than male samples in this collection. However, based on the age distribution, it is obvious that the sample's average age is in the 40s, and the upper limit is approximately 60. When it comes to hypertension, 0 means the individual does not have it, while 1 means the person has it. The total number of individuals who are healthy and have no history of heart disease is achieved in this dataset. With regard to BMI and average glucose levels, Figure 10 shows the relationship between one feature and the target feature.

Figure 10 shows the relationship between gender and stroke, age and stroke, hypertension and stroke, heart disease and stroke, ever_married and stroke, avg_glucose_level and stroke, and BMI and stroke.

### 3.2. Visualization of Feature Selection

The process of feature selection is shown in Figure 11. Feature selection aids in comprehending how features are linked to one another.

Figure 11 shows that age, hypertension, avg_glucose_level, heart_disease, ever_married, and BMI are positively corelated with the target feature. However, gender is negatively corelated with stroke.

### 3.3. Evaluation of the Model

#### 3.3.1. Random Forest (RF)

Figure 12 depicts the classification report for the RF model.

In this case, the total F1-score obtained is 96 percent. The individual F1-scores for healthy people are 96 percent, while those who have had a brain stroke have 96 percent. This model achieved the highest accuracy after fine-tuning. Prior to fine-tuning, the model had an accuracy of 92 percent.

Figure 13 depicts the random forest model's prediction. The predicted outcome and the model's calculated performance are shown in the confusion matrix. There are 2707 accurate guesses and 113 erroneous predictions.

#### 3.3.2. Decision Tree

The classification report for the decision tree classification is shown in Figure 14.

The final F1-score in this case is 94 percent. An individual's F1-score is 94 percent for healthy individuals and 95 percent for those who have had a brain stroke. Also, the precision and recall are shown in Figure 14. A fine-tuned decision tree model has also been implemented. However, after fine-tuning, the accuracy did not improve.

Figure 15 depicts the DT model's prediction. There were 2664 accurate guesses and 156 erroneous predictions.

#### 3.3.3. Voting Classifier

The classification report for the voting classifier is shown in Figure 16.

The total F1-score obtained in this case is 91 percent. The individual F1-scores are 91 percent for healthy people and 91 percent for those who have had a stroke. Also, the precision and recall are shown in Figure 16. Without any fine-tuning, this model achieved 91 percent accuracy.

The prediction made by the voting classifier is shown in Figure 17. The overall number of accurate guesses is 2565, while the total number of erroneous predictions is 255.

### 3.4. Model Comparison

Table 1 shows a comparison of the models with those found in prior studies. The chart clearly demonstrates that of the various models included in the framework, the RF model is the most effective. In addition to having a higher F1-score, it has more precision and better recall and accuracy.

From Table 1, it is clear that all algorithms have an acceptable level of accuracy, but the random forest algorithm is a preferable option because of its higher level of accuracy. This paper achieved 96 percent accuracy using the RF algorithm, but in [21] the authors achieved only 73 percent accuracy. Also, using the decision tree algorithm, this paper achieved 94 percent accuracy, while the authors in [21] achieved 77.6 percent accuracy. Although the KNN algorithm has not been implemented in this research, ref [12] achieved 95 percent accuracy, which is higher than the voting classifier's accuracy (91 percent). However, in this paper, logistic regression performs poorly.

## 4. Conclusion

Stroke is a life-threatening medical illness that should be treated as soon as possible to avoid further complications. The development of an ML model could aid in the early detection of stroke and the subsequent mitigation of its severe consequences. The effectiveness of several ML algorithms in properly predicting stroke based on a number of physiological variables is investigated in this study. Random forest classification outperforms the other methods tested with a classification accuracy of 96 percent. According to the research, the random forest method outperforms other processes when cross-validation metrics are used in brain stroke forecasting. The future scope of this study is that using a larger dataset and machine learning models, such as AdaBoost, SVM, and Bagging, the framework models may be enhanced. This will enhance the dependability of the framework and the framework's presentation. In exchange for just providing some basic information, the machine learning architecture may help the general public in determining the likelihood of a stroke occurring in an adult patient. In an ideal world, it would help patients obtain early treatment for strokes and rebuild their lives after the event.

## Figures and Tables

**Figure 1:** Proposed system's block diagram.

**Figure 2:** Total number of stroke and normal data.

**Figure 3:** Output column after preprocessing.

**Figure 4:** Block diagram of Random Forest Classifier.

**Figure 5:** Basic structure of a decision tree classifier.

**Figure 6:** Flowchart of a voting classifier.

**Figure 7:** Structure of a logistic regression classifier.

**Figure 8:** Block diagram of confusion matrix.

**Figure 9:** Histogram of some important features of the dataset.

**Figure 10:** Relationship between some important features with the target feature.

**Figure 11:** Features correlation with stroke.

**Figure 12:** Classification report of random forest.

**Figure 13:** Confusion matrix of random forest.

**Figure 14:** Classification report of decision tree.

**Figure 15:** Confusion matrix of a decision tree.

**Figure 16:** Classification report of a voting classifier.

**Figure 17:** Confusion matrix of a voting classifier.

**Table 1:** Performance comparison.

This paper (model name)	Accuracy (%)	Reference paper (model name)	Accuracy (%)
Random forest	96	Ref [21] random forest	73
Decision tree	94	Ref [21] decision tree	77.6
Voting classifier	91	Ref [12] K-nearest neighbor	95
Logistic regression	79	Ref [21] logistic regression	77.6

## Data Availability

The data utilized to support this research findings are accessible online at https://www.kaggle.com/fedesoriano/stroke-prediction-dataset.
